The article "The Role of Tomographic Ultrasonography in Conduit Mapping before Coronary Artery Bypass Grafting" was retracted in 2020. Reasons: no approval from the institution; copyright claims.

# The Role of Tomographic Ultrasonography in Conduit Mapping before Coronary Artery Bypass Grafting

**DOI:** 10.1155/2018/2097305

**Published:** 2018-11-21

**Authors:** Syed Mohammad Asim Hussain

**Affiliations:** Pennine Acute Foundation NHS Trust, UK

## Abstract

**Objective:**

To assess the performance of tomographic ultrasonography (TUS) in providing images that will enable optimum choice of vein segment to harvest for coronary artery bypass grafting (CABG).

**Methods:**

This was a prospective study of diagnostic accuracy. The index test was tomographic ultrasonography. The reference standard was intraoperative observation. The study was performed at the Vascular Imaging and Cardiothoracic Department at Wythenshawe Hospital, Manchester. Patients undergoing CABG who require vein mapping were included in the study. The main outcome measures were the number of tributaries identified in harvested vein segments, presence of varicosities, and usable length of vein.

**Results:**

The TUS correctly identified 89 out of 111 vein tributaries in 10 patients resulting in a sensitivity of 80.2%. This resulted in a p value of 0.000001 using an exact binomial test, with a prior probability of 0.5. TUS had a sensitivity of 66.7% and a specificity of 100% in the identification of varicosities over 14 patients. TUS had 90% agreement with intraoperative observation in assessing usable length of vein over 14 patients.

**Conclusions:**

Our results show that TUS has a high sensitivity in identifying vein tributaries. This can be used to select veins with fewer tributaries for harvesting should TUS be used for preoperative vein mapping before CABG.

## 1. Introduction

Coronary artery bypass grafting (CABG) is one of the most commonly performed cardiovascular operations. In the UK, approximately 20,000 procedures are completed annually at an estimated cost per capita of £8000 [1]. It is major surgery with a reported mortality of 1.08% in 2015 [1].

CABG surgery requires the use of arterial or venous conduits for revascularisation of diseased coronary arteries. The most commonly used conduits are the internal mammary artery (IMA) and great saphenous vein (GSV).

The GSV has historically been used for revascularisation of the right coronary artery and left circumflex artery and is the most commonly used conduit [2]. Its long length and ease of access makes it an ideal conduit choice.

### 1.1. Vein Quality

The ideal characteristics of a quality vein conduit have been extensively researched. They include having small number of tributaries and a diameter > 3mm that increases mildly and progressively from ankle to groin. There should be uniformity of calibre, no bifurcations, no varicosities, and no scarring from previous thrombophlebitis. Each of these factors is associated with saphenous vein flow and affects vein graft patency [3].

The article "The Role of Tomographic Ultrasonography in Conduit Mapping before Coronary Artery Bypass Grafting" was retracted in 2020. Reasons: no approval from the institution; copyright claims.

The GSV patency rate is not as high as arterial conduits such as the internal mammary artery or radial artery. Studies have shown that the patency rate of the GSV following CABG at 1 year is 80% which drops to 50% after 10 years [4]. Vein graft failure is associated with further revascularisation procedures, myocardial infarction, and death [5].

Vein graft failure can occur due to mechanical trauma during harvesting leading to graft ischaemia, endothelial damage, and turbulent flow [6]. Veins with more tributaries and varicosities are correlated with poor flow leading to an increased risk of graft failure. The vein can be damaged during the harvesting procedure by a number of mechanisms [6].

### 1.2. Role of Imaging

Preoperative vein mapping is used to facilitate GSV harvesting and reduce complications. Standard duplex ultrasonography (SDU) is the current imaging modality of choice and provides information regarding vein diameter and quality [7]. It has shown strong correlation with surgical measurements and can clearly demonstrate abnormalities in vein including areas of varicosity. It has resulted in significant reduction in incision length and harvest time which have improved postoperative recovery and reduced hospital stay [8]. However, it cannot identify tributaries which need to be identified and ligated.

Standard duplex ultrasound (SDU) provides a dynamic assessment at the time and requires ultrasound operators to build a three-dimensional mental impression of the vessel and vascular pathology. This process is highly operator dependent meaning scan quality is variable person to person. As a result, a level of understanding must exist between the ultrasound operator and surgeon, in identifying the optimum vessel. There is no facility to store the images for later viewing when using standard duplex ultrasonography.

### 1.3. Tomographic Ultrasonography

Tomographic ultrasonography (TUS) is a modified ultrasound technique which provides information in greater detail compared to SDU. The technology uses a tomographic laptop coupled to a regular ultrasound device to produce three-dimensional images. This technology is compatible with most commercially available ultrasound systems.

In our study, we used freehand 2D ultrasound scanners as they are flexible and convenient to operate. A wireless sensor was clipped into a regular ultrasound transducer to track the probe position. This obviated the need for an external position tracking system. Only a cable was required to connect the ultrasound transducer to a tomographic laptop. A digital video output was created which was processed by the tomographic laptop based on image reconstruction algorithms in order to produce a 3D volume.

The article "The Role of Tomographic Ultrasonography in Conduit Mapping before Coronary Artery Bypass Grafting" was retracted in 2020. Reasons: no approval from the institution; copyright claims.

Tomographic ultrasonography is less time-consuming than magnetic resonance imaging (MRI). It does not require nephrotoxic contrast like computed tomographic (CT) scans. Unlike SDU, it produces images that can be directly viewed by the surgeon. This allows a detailed preoperative assessment which should reduce graft complications.

The main benefit of tomographic ultrasonography is that it can reduce operator dependence and improve scan quality as the vessel is reconstructed into a three-dimensional image that can be manipulated to view the vessel from all angles. Galeandro et al. have previously reported that physicians with little vascular knowledge understand vein mapping better when demonstrated in a three-dimensional image [9].

Tomographic ultrasonography has already been shown to be an effective imaging modality in delineating foetal heart anatomy and assessing pelvic floor dysfunction. It is particularly useful for imaging the outflow tracts of the foetal heart which may be technically unfeasible with SDU [10]. It was able to demonstrate anatomical abnormalities in foetuses with pathologies such as Tetralogy of Fallot, Transposition of Great Vessels (TGV), and pulmonary stenosis in all cases [10]. In the assessment of pelvic floor, TUS allows a previously unattainable degree of quantification of levator-ani trauma [11]. Tomographic ultrasonography was found to have high repeatability, good generalisability, and a very low false-positive rate in a study assessing levator-ani avulsion [11].

In this study we will use TUS to map the GSV prior to CABG.

## 2. Hypothesis and Aims of Study

### 2.1. Aims

In studying whether tomographic ultrasonography is an adequate imaging modality for preoperative assessment of vascular conduits prior to coronary artery bypass grafting we seek to answer the following questions:

1. What is the sensitivity of TUS in identifying branches of the GSV?
2. What is the specificity of TUS in identifying a varicose GSV?

### 2.2. Hypothesis

Tomographic ultrasonography will provide preoperative images which will allow choice of optimum vein segment to harvest for CABG. An optimum vein segment is one with few tributaries. Additionally, it should have a diameter > 3mm, uniform calibre, and no varicosities or scarring due to thrombophlebitis.

## 3. Methods

### 3.1. Study Design

This was designed as a prospective study of diagnostic accuracy according to STARD 2015 guidelines [12]. We compared images of the Great Saphenous Vein acquired with tomographic ultrasound to intraoperative assessment under direct vision.

The article "The Role of Tomographic Ultrasonography in Conduit Mapping before Coronary Artery Bypass Grafting" was retracted in 2020. Reasons: no approval from the institution; copyright claims.

### 3.2. Subjects and Setting

This study occurred at the Cardiothoracic Department and the Vascular Studies Unit at Wythenshawe Hospital between January 2018 and March 2018. Consecutive eligible patients undergoing coronary artery bypass grafting who required vein mapping were enrolled in the study.

### 3.3. Inclusion Criteria

Patients undergoing coronary artery bypass grafting who require vein mapping.

### 3.4. Exclusion Criteria

Patients with the following factors are excluded as they complicate ultrasonographic assessment:

1. Immobility
2. Previously harvested saphenous veins
3. Unstable angina
4. Pacemakers
5. Positive microbiology and active infection

### 3.5. Study Intervention

TUS was performed with the patient standing as this optimises venous filling and visualisation. A tomographic computer was coupled to a high-end ultrasound scanner with a cable. The focus, depth, gain, colour scale, and colour gain were optimised. Once the leg was visualised without changing depth, a sweep was made and the TUS was activated to record.

A full-length image of the GSV was produced bilaterally with the location and number of tributaries marked for each vein segment. Specifically, the presence of varicosities, thrombophlebitis, and scarring was recorded. The usable length of vein was measured in centimetres and then divided by 18 cm. This is the standard length of Metzenbaum scissors which are used intraoperatively to determine vein length of one segment and is the approximate length of vein needed for one bypass graft.

A standard duplex ultrasound report was also written and placed in the patient notes. Surgery was later performed with the standard duplex report available. The TUS report was not shown to the vein harvester before the operation.

The reference standard was intraoperative measurement of the above variables. The number of tributaries seen in the harvested vein was counted and recorded. The usability of vein segments was determined using standard length of Metzenbaum scissors (18 cm = 1 segment of vein). A vein segment was considered usable if it had the following: a diameter > 3 mm upon inflation with blood or saline but < 5mm, uniform calibre, and no varicosities, thrombophlebitis, or scarring. The diameter was measured at the divided distal end of the vein using forceps and sterile tape measure.

### 3.6. Blinding

This was a single blind study. Reference standard results were not available to the radiographer performing the index test. Index test results were not available to the vein harvester. Two experienced vein harvesters observed the number of tributaries and varicosities intraoperatively. Two experienced radiographers analysed the ultrasonographic data.

The article "The Role of Tomographic Ultrasonography in Conduit Mapping before Coronary Artery Bypass Grafting" was retracted in 2020. Reasons: no approval from the institution; copyright claims.

The data was documented at the time of surgery and the vein harvesters' and radiographers' did not participate in subsequent data analysis. This prevented the analysis from being influenced through anecdotal evidence derived from the vein harvester or radiographers personal experience of TUS.

### 3.7. Outcome Measures

The endpoints for the study are stated below.

1. Number of tributaries in harvested vein segments and corresponding segments on TUS. An exact binomial test and agreement analysis was performed
2. Presence of varicosities on TUS and intraoperatively. Sensitivity and specificity of TUS in identifying varicosities
3. Usable length of vein as measured intraoperatively and on tomographic ultrasonography. An agreement analysis was performed

A standardised form was filled by the vein harvesters and radiographers. Academic interest was in the presence of varicosities rather than the exact number and whether the diameter was between 3 and 5 mm rather than an exact value. We were primarily interested in the number of vein tributaries and vein usability.

## 4. Ethics Approval

Ethics approval was granted on 28/4/2016 by the North West-Greater Manchester and South Research Ethics Committee. REC reference is 16/NW/0153.

## 5. Ethics, Consent, and Permissions

All participants gave written consent to participate in the study.

## 6. Consent to Publish

I have obtained consent to publish from the participants.

## 7. Results

Nineteen patients were initially consented into the study. The demographic details are shown in Table 1. Out of these, 14 patients met the inclusion criteria and underwent a tomographic ultrasound scan, i.e., a proportion of 73.7%.

There were 11 male and 3 female patients in the study. The mean age was 66.6 years.

The total number of usable vein (Table 2) segments determined intraoperatively in fourteen patients was 28. The number of usable vein segments as determined by TUS was 33.

The mean difference (bias) was** 0.286** vein segments. The 95% CI upper limit of agreement was determined to be** 1.246** and the 95% CI lower limit of agreement was** -0.674.** Only one out of fourteen values fell outside the upper limit of agreement. This gives a percentage agreement of 92.3% within the 95% limits of agreement.

In our study of 14 patients, 3 had varicosities as determined by intraoperative observation, i.e., true positives (Table 3). The TUS was able to pick up 2 of these varicosities resulting in a sensitivity of** 66.7**%. The remaining 11 patients had normal veins and this was correctly identified by TUS in all 11 cases resulting in a specificity of** 100**%. 

The article "The Role of Tomographic Ultrasonography in Conduit Mapping before Coronary Artery Bypass Grafting" was retracted in 2020. Reasons: no approval from the institution; copyright claims.

Our primary endpoint was the sensitivity of TUS in identifying GSV tributaries. We compared 10 out of 14 samples. The number of vein tributaries in these 10 samples was** 111** as determined from intraoperative counting (Table 4). The number of vein tributaries as determined by tomographic ultrasonographic analysis was** 89. **This results in a sensitivity of** 80.2**%. An exact binomial test was performed assuming a neutral prior probability,* p* of 0.5, K of 89, and* n* of 111. This gives a one-tailed probability of exactly, or greater than, 89(K) out of 111(n) of ***p *< 0.000001. **

An agreement analysis was performed between TUS and intraoperative observation in determining GSV tributaries. The bias (mean difference) was equal to** -2.2**. The 95% CI upper and lower limit of agreement was** + 2.4** and** – 6.8,** respectively. Only one value was outside the lower limit of agreement. This gives an agreement of 90% within the limits of agreement.

A regression analysis was also performed. The correlation coefficient** r** was found to be** 0.77592**. The coefficient of determination **r**^2^ was found to be** 0.60205.**

The mean time taken to perform a tomographic ultrasound scan for both legs was 5 minutes. The mean time taken to perform a standard duplex ultrasound scan was 20 minutes.

Figure 1 shows the GSV as viewed from a tomographic ultrasound scanner. The image has been reconstructed to give a three-dimensional view allowing visualisation of tributaries.

## 8. Discussion

This study compared the performance of a new imaging modality, tomographic ultrasonography, against a reference standard provided by direct intraoperative observation across a range of parameters affecting vein graft quality.

### 8.1. Interpretation of Data

Our primary endpoint was the number of GSV tributaries correctly identified. To provide a fair comparison, we had to ensure that both the radiographer and the vein harvester were observing the same length of vein from the same anatomical location. Therefore, we excluded four results in which the radiographer may have been observing a larger length of vein which would have biased the result in favour of TUS.

TUS performed well correctly identifying vein tributaries with a sensitivity > 80%. This produced a highly statistically significant result (p < 0.000001) using an exact binomial test when compared with a prior probability null hypothesis of 0.5.

We performed a multivariate regression analysis to evaluate the role of confounding variables. The independent variables were intraoperative measurements. The correlation coefficient,** r,** was 0.77592 and the coefficient of determination, **r**^2^, was 0.60205 indicating that intraoperative measurements correlated well with tomographic ultrasonographic measurements.

The article "The Role of Tomographic Ultrasonography in Conduit Mapping before Coronary Artery Bypass Grafting" was retracted in 2020. Reasons: no approval from the institution; copyright claims.

We considered identification of varicose veins to be important. Extensive varicosities involving the GSV preclude its use as a conduit. This is because of their large, irregular diameter and thin walls. This will result in greater diameter mismatch with the host artery resulting in shear forces leading to endothelial damage. They are also more prone to phlebitis and thrombosis.

In our study, true varicose veins were diagnosed by tomographic ultrasonography 2 out of 3 times yielding a sensitivity of 66.7%. TUS correctly identified healthy, nonvaricose veins in all 11 cases resulting in a specificity of 100%.

Vein diameter and luminal irregularities are important factors in vein graft failure. The foremost pathological mechanism is focal intimal hyperplasia. Luminal irregularities can cause eddy currents associated with low shear stress and high shear gradients leading to focal intimal hyperplasia [13]. The damage to graft endothelium causes local release of tissue factors which contribute to thrombosis [14]. These mechanisms underscore the importance of a uniform calibre vessel.

One study analysed vein graft samples from 200 patients. It concluded that distinct irregularities result from an uneven distribution of side branches and that an average saphenous vein encounters 1.9 diameter changes of 20% and 1.2 diameter changes of up to 40% [15]. This suggests that a fewer number of vein tributaries would be associated with reduced turbulence and more uniform calibre.

Prior phlebitis precludes the use of the GSV as a conduit. This normally results in scarring that can make it technically difficult to harvest the vein. The inflammation can damage the vein wall and endothelium increasing the risk of thrombosis.

In our study, there were no patients with obvious vein abnormalities such as scarring or thrombophlebitis. Our results showed good agreement between TUS and intraoperative observation with regard to vein usability.

The total number of usable vein segments measured on TUS is 33 compared to 28 measured intraoperatively from 14 patients.

We observed that the mean time taken to perform a tomographic ultrasound scan on both legs was only five minutes while standard duplex ultrasonography took 20 minutes to perform. This is a significant benefit of tomographic ultrasonography in that it can be performed much faster. It also requires less expert personnel to perform this scan as the image reconstruction is done automatically. This has the potential to reduce cost and waiting lists for ultrasound scans.

The article "The Role of Tomographic Ultrasonography in Conduit Mapping before Coronary Artery Bypass Grafting" was retracted in 2020. Reasons: no approval from the institution; copyright claims.

### 8.2. Limitations of the Study

There were some limitations in our study. The most obvious one is the small sample size of 14 patients. This gives a post hoc statistical power of 38.2% at the 5% significance level assuming a null hypothesis of 50% tributaries correctly identified. A sample size of 38 patients would have given 80% power given the proportion of tributaries correctly identified by tomographic ultrasonography in this study. This prevents us from drawing significant conclusions although we are encouraged by the performance of TUS based on preliminary results. We would expect it to meet the 80% statistical power threshold with a larger sample size as the effect size is considerable.

The second limitation is the lack of randomisation and double blinding in this study. In ideal circumstances, it should not have been possible for the radiographer, vein harvester, or researcher to tell which patients are participating in the study.

The third limitation is the lack of standardisation in reporting by the two radiographers and the two vein harvester's potentially increasing interrater variability.

### 8.3. Future Perspectives

Despite these limitations, the study did provide useful information. This was particularly true for the sensitivity of TUS in identifying vein tributaries and generally good agreement with intraoperative observation. Preoperative vein mapping with TUS is likely to make the procedure of vein harvesting easier, quicker, and less traumatic.

Additionally, it will allow clinicians to select the optimum vein segment to harvest depending on how many tributaries can be visualised on TUS preoperatively. Choosing a vein segment with fewer tributaries can potentially reduce the incidence of saphenous vein graft failure. Such a segment would have a more uniform calibre and will generate less turbulence and haemodynamic stresses. This could potentially lead to a reduction in repeat revascularisation, myocardial infarction, and mortality.

It is important to note that this is a new imaging modality. With time, there are likely to be advancements in technology and reduction in cost. Therefore, the sensitivity of TUS in identifying vein tributaries should improve further.

TUS is also likely to fit in well with new strategies in care delivery for cardiovascular disease that aim to maximize patient choice. This is most evident in Project Leonardo which evaluated the feasibility and effectiveness of a new care management model that used care managers to liaise between patients, family physicians, and specialists to treat patients with cardiovascular disease, heart failure, and diabetes [16]. The project was highly effective in increasing patient health knowledge, self-management skills, and readiness to make changes in health [16]. TUS empowers patients further by providing an alternative to standard duplex imaging.

The article "The Role of Tomographic Ultrasonography in Conduit Mapping before Coronary Artery Bypass Grafting" was retracted in 2020. Reasons: no approval from the institution; copyright claims.

This was a novel study as TUS has not been used for conduit mapping for CABG before. We see potential in tomographic ultrasonography as an alternative to current preoperative vein mapping with SDU. Given the prevalence of CABG surgery, replacing SDU as the standard tool for vein mapping is likely to have a significant economic impact.

The next step is a large randomised trial comparing outcomes using both TUS and SDU for preoperative vein mapping. The endpoint should focus on both immediate and postoperative morbidity and longer-term effects on graft patency, myocardial infarction, and death.

## 9. Conclusion

Our study has shown that tomographic ultrasonography can identify vein tributaries with a high sensitivity and it correlates well with intraoperative observation. It has obvious advantages over standard duplex imaging in that it can be performed faster and requires less expert personnel.

## Figures and Tables

**Figure 1:** The great saphenous vein as seen with a 3D tomographic ultrasound scanner.

**Table 1:** Data showing demographic information, type of operation, and risk factors for cardiovascular disease in patients included in our study.

Age	Gender	Operation	Risk factors
49	Male	CABGx4	Hypertension, High Cholesterol, Ex-smoker
74	Male	CABGx4	Hypertension, High Cholesterol, Ex-smoker
73	Male	CABGx3	Hypertension, High Cholesterol, Ex-smoker
58	Male	CABGx3	Hypertension, High Cholesterol, Ex-smoker, positive family history
58	Female	CABGx3	Hypertension, High Cholesterol
63	Male	CABGx4	Hypertension, High Cholesterol, Smoker
61	Male	CABGx2+AVR	Hypertension, High Cholesterol, Ex-smoker, Type 2 Diabetes
53	Female	CABGx3	Hypertension, High Cholesterol, Ex-smoker, Type 2 Diabetes
74	Male	CABGx3	Hypertension, High Cholesterol
74	Male	CABGx4	Hypertension, High Cholesterol
73	Male	CABGx3	Hypertension, High Cholesterol, Ex- smoker
76	Male	CABGx4	Hypertension, High Cholesterol, Ex-smoker,
71	Male	CABGx3	Hypertension, High Cholesterol, Ex-smoker
76	Female	CABGx3	Hypertension, High Cholesterol

CABG: coronary artery bypass grafting, AVR: aortic valve replacement.

**Table 2:** This table shows usable vein segments determined by each measurement method.

TUS usable vein lengths	Intra-operative usable vein lengths	Mean of both measures	Difference of both measures
2	2	2	0
3	3	3	0
2	2	2	0
2	1	1.5	1
3	2.5	2.75	0.5
3	3	3	0
2	2	2	0
3	1.5	2.25	1.5
2	2	2	0
2	2	2	0
1	0	0.5	1
3	3	3	0
1	1	1	0
3	3	3	0
Total=33	Total=28		Mean difference=0.286

**Table 3:** This table shows sensitivity and specificity of TUS in identifying varicose veins.

**Tomographic ultrasound**	**Intra-operative observation**	
	**Varicosities**	**Normal veins**
**Positive**	2	0
**Negative**	1	11

The article "The Role of Tomographic Ultrasonography in Conduit Mapping before Coronary Artery Bypass Grafting" was retracted in 2020. Reasons: no approval from the institution; copyright claims.

**Table 4:** This table shows number of tributaries identified by each measurement method.

**TUS: Number of GSV tributaries**	**Intra-operative observation: Number of GSV tributaries**	**Mean of both methods**	**Difference between both methods**
**11**	13	12	-2
**12**	12	12	0
**10**	10	10	0
**14**	15	14.5	-1
**8**	15	11.5	-7
**9**	10	9.5	-1
**6**	6	6	0
**10**	15	12.5	-5
**2**	5	3.5	-3
**7**	10	8.5	-3
**Total = 89**	**Total = 111**		**Mean difference = -2.1**

## Data Availability

The data used to support the findings of this study are available from the corresponding author upon request.
